The article "lncRNA TINCR sponges miR-214-5p to upregulate ROCK1 in hepatocellular carcinoma" was retracted in 2021. Reasons: signs of a paper mill; lack of ethics approval or compliance.

# lncRNA TINCR sponges miR-214-5p to upregulate ROCK1 in hepatocellular carcinoma

**DOI:** 10.1186/s12881-019-0940-6

**Published:** 2020-01-03

**Authors:** Min Hu, Yaowu Han, Ying Zhang, Yuanfeng Zhou, Lin Ye

**Affiliations:** 1 Department of Pathology, Anhui University of Chinese Medicine, Hefei, 1 Qianjiang Road, Hefei, 230012 Anhui province China; 2 Graduate School, Anhui University of Chinese Medicine, Hefei, 230038 Anhui China; 3 Department of Psychology, Anhui University of Chinese Medicine, Hefei, 230012 Anhui China

**Keywords:** Hepatocellular carcinoma, lncRNA TINCR, miR-214-5p, ROCK1

## Abstract

**Background:**

Our preliminary bioinformatics analysis showed that lncRNA TINCR may absorb miR-214-5p by serving is sponge, while miR-214-5p targets ROCK1. This study aimed to investigate the interactions among these 3 factors in hepatocellular carcinoma (HCC).

**Methods:**

Expression of TINCR, ROCK1 and miR-214-5p in HCC and non-tumor tissues was detected by performing qPCR. The correlations among TINCR, ROCK1 and miR-214-5p in HCC tissues were analyzed by performing linear regression. Overexpression experiments were performed to analyze gene interactions. Cell proliferation was analyzed by CCK-8 assay.

**Results:**

We found that TINCR and ROCK1 were upregulated, while miR-214-5p was downregulated in HCC. TINCR and ROCK1 were positively correlated, while TINCR and miR-214-5p were not significantly correlated. In HCC cells, TINCR overexpression is followed by ROCK1 overexpression, while miR-214-5p overexpression induced the downregulation of ROCK1. In addition, TINCR and miR-214-5p did not affect the expression of each other. TINCR and ROCK1 overexpression led to increased rate of cancer cell proliferation, while miR-214-5p played an opposite role and reduced the effects of TINCR overexpression. Therefore, TINCR sponges miR-214-5p to upregulate ROCK1 in HCC, thereby promoting cancer cell invasion and migration.

## Background

Incidence of hepatocellular carcinoma (HCC) ranks top places all over the world [1]. With the popularization of risk factor screening program and the application of prevention regimens, incidence of HCC has dropped significantly in many regions, such as parts of China and Japan [2]. However, an increasing trend in both incidence and mortality rates of HCC has been observed in many European countries and North America owing to the high prevalence of hepatitis B virus (HBV) and hepatitis C virus (HCV) infections [3]. In spite of the considerable number of risk factors identified for HCC, pathogenesis of this disease remains poorly understood [4, 5], which is a big challenge in the development of novel therapeutic targets.

ROCK1, or Rho-associated protein kinase 1, acts at the downstream of small GTPase RhoA to mediate the formation of contractile force [6]. Oncology studies have shown that ROCK1 is usually overexpressed during cancer development and ROCK1 overexpression promotes cancer development by regulating cancer cell behaviors, such as proliferation, invasion and migration [7, 8]. In effect, inhibition of ROCK1 is novel therapeutic choice for cancer [7, 8]. It is known that, the expression of ROCK1 can be regulated by certain miRNAs [9, 10], and the function of miRNAs can be attenuated by lncRNA sponges [11]. In a recent study, Zhang et al. reported that miR-214-5p inhibits osteosarcoma cell proliferation by directly targeting ROCK1 [12]. TINCR has been reported to be an oncogenic lncRNA in many types of cancers including HCC [13]. Our bioinformatics analysis showed that TINCR may sponge miR-214-5p. This study was performed to investigate the interactions among TINCR, miR-214-5p and ROCK1 in HCC.

## Methods

### Patients and specimens

Form December 2016 to December 2018 a total of 137 HCC patients were admitted by Anhui University of Chinese Medicine. From those patients our study selected 60 cases (gender: 37 males and 23 females; age: 33 to 67 years; mean: 49.9 ± 6.3 years) to serve as research subjects. Inclusion criteria: 1) No therapies for any clinical disorders were performed within 100 days; 2) new HCC cases. Exclusion criteria: 1) patients with other clinical disorders; 2) patients with recurrent HCC; 3) patients with previous history of malignancies. The HCC patients were educated with the experimental principle and all of them involved in this study provided signed informed consent. All patients were diagnosed by histopathological biopsy. During the operation of biopsy, non-tumor and HCC tissues were collected from each patient. All tissue specimens were confirmed by at least 3 experienced pathologists. This study has been approved by Ethics Committee of Anhui University of Chinese Medicine.

### HCC cells and transient transfections

In vitro experiments in this study were performed using HCC cell lines H1581 (Cat# ATCC® CRL-5878™) and SNU-475 (ATCC® CRL-2236™) from ATCC (USA). Cells were cultivated at 37 °C with 5% CO_2_ in RPMI-1640 medium (10% FBS) before use. PcDNA3.1 vectors expressing TINCR and ROCK1 were constructed by RIBOBIO (Guangzhou, China). MiR-214-5p mimic and negative control miRNA were also from RIBOBIO. H1581 cells were harvested and were counted, followed by transfection of 10 nM pcDNA3.1 vector expressing TINCR or ROCK2, or 10 nM empty pcDNA3.1 vector (negative control, NC), or 30 nM miR-214-5p mimic, or 30 nM negative control miRNA (NC) into 10^6^ cells through lipofectamine 2000 (Invitrogen, USA)-mediated method. Cells with no transfections were also included to serve was control (C) group. The interval between subsequent experiments and transfection was 24 h.

### RNA extractions and qPCR

Non-tumor and HCC tissues were ground. H1581 cells were harvested and counted. To extract total RNAs, 0.015 g tissue or 10^6^ cells were mixed with 1 ml Trizol reagent (Invitrogen, USA). To retain miRNA, 80% ethanol was used to participate and wash RNAs. MMLV Reverse Transcriptase (Lucigen, USA) and QuantiTect SYBR Green PCR Kit (Qiagen, Shanghai, China) were used to perform total RNA reverse transfections and prepare qPCR mixtures to detect the expression of TINCR and ROCK2 with GAPDH as endogenous control. miScript II RT Kit (QIAGEN) and miScript SYBR Green PCR Kit (QIAGEN) were used to perform miRNA reverse transcriptions and prepare qPCR mixtures to detect the expression of miR-214-5p with U6 as endogenous control. All experiments were performed in triplicate manner and expression levels were normalized using 2^-ΔΔCT^ method.

### Western blot analysis

H1581 cells were collected and mixed with RIPA solution (RIBOBIO) with a ratio of 10^5^ cells per 1 ml solution. Total proteins were extracted following the protocol provided by RIBOBIO. Protein samples were quantified using BCA kit (RIBOBIO), followed by denaturing in boiled water for 5 min. Following 12% SDS-PAGE gel electrophoresis, gel transfer (PVDF membrane) and blocking (2 h in 5% non-fat milk at room temperature) were performed. Following that, primary antibodies of rabbit GAPDH (1: 1500, ab37168, Abcam) and RCOK1 (1: 1200, ab66320, Abcam) were used to blot the membranes at 4 °C for 15 h. After that, HRP goat anti-rabbit (IgG) secondary antibody (1:1400; ab6721; Abcam) was used to further blot the membranes for 2 h at 24 °C. All signal developments were performed using ECL solution (Sangon, Shanghai, China). Image J v1.46 software was used to normalize all gray values.

### RNA-RNA interaction prediction

The interaction between TINCR and miR-214-5p was performed using online program IntaRNA (http://rna.informatik.uni-freiburg.de/IntaRNA/Input.jsp). Sequence of TINCR was used as the long sequence and sequence of miR-214-5p was used as the short sequence. All other parameters were default.

### Cell proliferation analysis

H1581 and SNU-475 cells were harvested and counted. 1 ml RPMI-1640 medium (10% FBS) was mixed with 5 × 10^4^ cells to prepare single cell suspensions. The cells were cultivated in a 96-well plate (0.1 ml per well) at 37 °C in a 5% CO_2_ incubator. Three replicate wells were set for each experiment. To monitor cell proliferation, 10ul CCK-8 solution (Sigma-Aldrich) was added at 2 h before the end of cell culture. Cell collection was performed every 24 h for a total of 4 days. After the termination of cell culture OD values at 450 nm were measured. OD value of Control group was set to “100”, all other time pointes and other groups were normalized to this value.

### Statistical analysis

Data from 3 biological replicates were used to calculate mean values, which were used in all data analyses. Correlations were analyzed by linear regression. Differences in gene expression levels and cell proliferation rates among aforementioned different cell transfection groups were analyzed by ANOVA (one-way) and post hoc Tukey test. Differences in levels of gene expression between non-tumor and HCC tissues were explored using paired t test. With the median expression level of TINCR in HCC as cutoff value, the 60 patients were divided into high and low TINCR level group (*n* = 30). Chi-squared test was performed to analyze the relationship between patients’ clinical data and levels of TINCR expression in HCC. *p* < 0.05 was statistically significant.

## Results

### Expression of TINCR, ROCK1 and miR-214-5p was altered in HCC

Expression of TINCR, ROCK1 and miR-214-5p in HCC and non-tumor tissues was detected by performing qPCR. Expression levels were compared between non-tumor and HC tissues by paired t test. Compared to non-tumor tissues, expression levels of TINCR (Fig. 1a) and ROCK1 (Fig. 1b) were significantly higher, whereas expression level of miR-214-5p was significantly lower (Fig. 1c) in HCC (*p* < 0.05). Chi-squared test showed that levels of TINCR in HCC tissues were significantly correlated with tumor size and TNM stage (*p* < 0.05), but not age, gender, histological differentiation, HBV or HCV infections and liver cirrhosis (*p* < 0.05, Table 1).

**Fig. 1:** Expression of TINCR, ROCK1 and miR-214-5p was altered in HCC. Expression of TINCR (**a**), ROCK1 (**b**) and miR-214-5p (**c**) in HCC and non-tumor tissues was detected by performing qPCR. All qPCR reactions were performed 3 times. Expression levels were compared between non-tumor and HC tissues by paired t test (*, *p* < 0.05)

**Table 1:** Correlation between levels of TINCR expression levels in HCC and patients’ clinical data

Variables	n	High (*n* = 30)	Low (*n* = 30)	Chi square	p
Gender					
Male	37	17	20	0.63	0.43
Female	23	13	10		
Age (years)					
> 50	28	13	15	0.27	0.60
< =50	32	17	15		
Histological differentiation					
Well	14	5	9	1.55	0.46
Moderate	21	11	10		
Poor	25	14	11		
HBV or HCV infections					
Yes	48	22	26	1.67	0.20
No	12	8	4		
Liver cirrhosis					
Absence	11	5	6	0.11	0.74
Presence	49	25	24		
Tumor size					
> 5 cm	33	10	23	11.38	0.0007
< = 5 cm	27	20	7		
TNM stage					
I + II	31	11	20	5.41	0.02
III + IV	29	19	10		

### The correlations among TINCR, ROCK1 and miR-214-5p in HCC

The correlations among TINCR, ROCK1 and miR-214-5p in HCC tissues were analyzed by performing linear regression. In HCC tissues, TINCR and ROCK1 were positively correlated (Fig. 2a), while TINCR and miR-214-5p were not significantly correlated (Fig. 2b). In addition, miR-214-5p and ROCK1 were also not significantly correlated (Fig. 2c).

**Fig. 2:** The correlations among TINCR, ROCK1 and miR-214-5p in HCC. The correlations between TINCR/ROCK1 (**a**), TINCR/miR-214-5p (**b**) and miR-214-5p/ROCK1 (**c**) were analyzed by linear regression

### TINCR may sponge miR-214-5p

The interaction between TINCR and miR-214-5p were predicted using the aforementioned methods. It can be observed that TINCR may form base pairing with miR-214-5p from position 258 to position 276 (Fig. 3). The hybridization energy is − 22.7 kcal/mol. Therefore, TINCR can be a sponge of miR-214-5p.

**Fig. 3:** TINCR may sponge miR-214-5p. The interaction between TINCR and miR-214-5p was performed using online program IntaRNA. Sequence of TINCR was used as the long sequence and sequence of miR-214-5p was used as the short sequence. All other parameters were default

### The interactions among TINCR, ROCK1 and miR-214-5p in H1581 cells

TINCR and ROCK1 expression vectors as well as miR-214-5p mimic were transfected into H1581 cells. At 24 h post-transfection, expression levels of TINCR, ROCK1 and miR-214-5p were significantly upregulated Compared to NC and C groups (Fig. 4a, *p* < 0.05). In addition, TINCR overexpression is followed by ROCK1 overexpression, while miR-214-5p overexpression induced the downregulation of ROCK1 and attenuated the effects of ROCK1 overexpression (Fig. 4b, *p* < 0.05). In addition, TINCR and miR-214-5p did not affect the expression of each other (Fig. 4c).

**Fig. 4:** The interactions among TINCR, ROCK1 and miR-214-5p in HCC cells. TINCR and ROCK1 expression vectors as well as miR-214-5p mimic were transfected into H1581 cells. At 24 h post-transfection, overexpression of TINCR, ROCK1 and miR-214-5p was confirmed by qPCR (**a**). The effects of TINCR and miR-214-5p on ROCK1 overexpression were analyzed by qPCR and western blot (**b**). The interaction between TINCR and miR-214-5p was analyzed by qPCR (**c**). All experiments were repeated 3 times and mean values were presents. NC1, empty vector transfection; NC2, negative control miRNA transfection (*, *p* < 0.05)

### TINCR promoted H1581 and SNU-475 cell proliferation through ROCK1 and miR-214-5p

Cell proliferation data were analyzed. Compared to C and NC groups, TINCR and ROCK1 overexpression led to increased rate of cancer cell proliferation, while miR-214-5p played an opposite role and reduced the effects of TINCR overexpression (Fig. 5, *p* < 0.05).

**Fig. 5:** TINCR promoted HCC cell proliferation through ROCK1 and miR-214-5p. The effects of TINCR, ROCK1 and miR-214-5p on HCC cell proliferation were analyzed by cell proliferation assay. All experiments were repeated 3 times and mean values were presents. NC1, empty vector transfection; NC2, negative control miRNA transfection (*, *p* < 0.05)

## Discussion

This study mainly investigated the interactions among TINCR, ROCK1 and miR-214-5p in HCC. We found that TINCR can upregulate ROCK1 possibly by sponging miR-214-5p, which can directly target ROCK1.

Previous studies have identified numerous miRNAs that can directly target ROCK1 [9, 10, 12]. In HCC, miR-148b targets ROCK1 to inhibit cancer cell proliferation, invasion and migration [14]. In a recent study, miR-214-5p was reported to directly target ROCK1 to inhibit cancer cell behaviors [12]. In the present study we also observed the reduced expression levels of ROCK1 in HCC cells after miR-214-5p expression. Therefore, miR-214-5p may also target ROCK1 to regulate its expression in HCC. Those data also suggest that ROCK1 can be targeted by multiple miRNAs.

In this study we observed the upregulated ROCK1 and downregulated miR-214-5p in HCC tissues. Interestingly, we did not observe a significant correlation between miR-214-5p targets ROCK1 in HCC tissues. This observation suggests the existence of a sponge of miR-214-5p. MiRNA sponges only absorb miRNAs to attenuate their functions but may not affect their expression levels [15]. Therefore, if a sponge exists, the downregulation of miR-214-5p expression may not be significantly correlated with the upregulated ROCK1. The sponge may serve buffer to finely regulate the levels of functional miRNAs.

TINCR is a well-characterized oncogenic lncRNA in many types of cancer [13, 16, 17]. In some cases, TINCR may sponge miRNAs to promote cancer progression. For instance, TINCR sponges miR-375 to regulate PDK1, thereby promoting gastric cancer [16]. In colorectal cancer, TINCR sponges miR-7-5p to aggregate disease conditions [17]. In this study we showed that TINCR may sponge miR-214-5p to upregulated ROCK1 in HCC, and the upregulation of ROCK1 by TINCR is involved in the regulation of HCC cell proliferation. However, other lncRNAs may also sponge miR-214-5p to participate in this process. Our future studies will explore this possibility.

## Conclusions

In conclusion, TINCR played an oncogenic role in HCC by sponging miR-214-5p to upregulate ROCK1.

## Data Availability

The analyzed data sets generated during the study are available from the corresponding author on reasonable request.

## Abbreviations

FBS: Fetal bovine serum
GAPDH: Glyceraldehyde 3-phosphate dehydrogenase
HBV: Hepatitis B virus
HCC: Hepatocellular carcinoma
HCV: Hepatitis C virus
ROCK1: Rho Associated Coiled-Coil Containing Protein Kinase 1
TINCR: TINCR ubiquitin domain containing
